The article "An Exploratory Study on the Relationship between Brachial Arterial Blood Flow and Cardiac Output" was retracted in 2023. Reasons: unreliable results or conclusions; concerns about the data; concerns about the peer review; concerns about the citations.

# An Exploratory Study on the Relationship between Brachial Arterial Blood Flow and Cardiac Output

**DOI:** 10.1155/2021/1251199

**Published:** 2021-12-23

**Authors:** Sixiang Jia, Yiteng Wu, Wei Wang, Wenting Lin, Yiwen Chen, Huanyu Zhang, Shudong Xia, Hong Zhou

**Affiliations:** ^1^Department of Heart Center, The Fourth Affiliated Hospital of Zhejiang University School of Medicine, N1 Shangcheng Road, Yiwu 322000, China; ^2^College of Biomedical Engineering & Instrument Science, Zhejiang University, Hangzhou 310000, China

## Abstract

**Background:**

We have obtained prospective clinical outcomes using the brachial artery largely, such as Korotkoff sound and vasomotor function measurement by ultrasound guidance to predict the prognosis of cardiovascular diseases. Very few reports on the quantitative measurement of the relationship between the brachial artery blood flow and cardiac output have been reported.

**Purpose:**

(1) To investigate whether the quantitative relationship between the brachial artery blood flow and cardiac output existed. (2) To provide a theoretical basis for taking advantage of artificial intelligence (AI) using Korotkoff sound analogously as far as possible to predict the cardiac output.

**Methods:**

A total of 586 patients who underwent cardiac color ultrasound in our center from 2021.3 to 2021.7 were included for analyses. The vascular parameters of the right upper limb brachial artery (such as the Diameter, Area, Blood Velocity, and Flow) were measured immediately after the cardiac color ultrasound, and some basic clinical parameters (Age, Sex, BMI, and Disease) were recorded subsequently. Ultimately, the Mann–Whitney and independent sample *T*-test were used to analyze the data.

**Results:**

(1) The mean Rate of the brachial arterial blood flow to cardiac output was 1.23%, and the mean 95% CI was (1.18%, 1.29%), indicating that the value was mainly concentrated in the current value interval. The indicator demonstrates that there is no significant difference currently among the patients with hypertension, coronary heart disease, and cardiac dysfunction. (2) The brachial artery wall diameter (Dist) is significantly thicker in patients with coronary heart disease and hypertension compared to patients with other cardiovascular diseases. (3) Cardiac output augments remarkably in patients with hypertension.

**Conclusion:**

Our study suggests that the Rate (brachial artery blood flow/cardiac output) is a constant of 1.23% approximately. It provides a theoretical basis for the subsequent application of the artificial intelligence (AI) method to predict heart function using Korotkoff sound, cope with large computational amounts, and improve computational speed. It is also indirectly proved that hypertension can lead to a change in peripheral vascular hyperplasia and increase cardiac output.

## 1. Introduction

Chronic heart failure (CHF) is the terminal stage of most patients with cardiovascular disease, and the prognosis is often poor. Traditional risk factors incompletely predict the development of cardiovascular disease, which is often the leading cause of cardiovascular death worldwide [1]. Our research team has been working on nondestructive methods for early and accurate identification of the signals of cardiovascular disease progression. Korotkoff sound is a hot research topic based on the objective of the brachial artery in the cardiovascular field all the time [2]. Domestic and foreign scholars have studied the brachial artery exploiting the mechanism of Korotkoff sound and obtained fruitful prospective results, which are as follows: (1) the QKD method based on the pulse wave theory [3] and (2) the AVI method based on pulse pressure, etc. [4]. To date, there are few reports on the correlation between Korotkoff sound's signal characteristics and cardiovascular diseases.

In 2002, Corretti et al. used the endothelium-dependent flow-mediated vasodilation (FMD) technique to measure the flow and velocity of the brachial artery by ultrasound, indirectly proving the correlation between the degree of brachial artery endothelial dilation and the development of hypertension or coronary heart disease [5]. However, its specific mechanism has not been clarified in detail, pending a follow-up and an in-depth study. Now, with the efforts of continuous exploration, domestic and foreign scholars preliminarily determined that the Korotkoff sound is caused by the blood turbulence triggering the brachial artery wall vibration [6]. Based on the mechanism of Korotkoff sound, it can be inferred that when the patient's cardiac ejection capacity reduces, the blood flow through the brachial artery per unit time will decrease accordingly, leading to the transformation of the impact force and blood flow velocity on the blood vessel wall and to the influencing of the characteristics of Korotkoff sound signal. We have not known how the brachial artery blood flow and cardiac output alternation are detailed according to the current paper yet.

From the perspective of the relationship between the brachial artery blood flow and cardiac output, this study, if successful, will provide a theoretical basis for the subsequent use of artificial intelligence (AI) to predict cardiac output by Korotkoff sound method and optimize the data volume to a certain extent. So far, few similar studies have been reported. The following are the major contributions of this paper:

1. To explore whether there would be a quantitative relationship between the brachial arterial blood flow and cardiac volume in patients (Rate = Brachial arterial blood flow/Cardiac Output) and whether these the Rate would be more outstanding in patients with cardiac dysfunction.
2. The secondary outcome was to explore whether the brachial artery diameter (Dist), blood flow (Vol Flow), and Cardiac Output in the patients with different cardiovascular diseases having otherness.
3. In the statistical analysis of differences, to study the differences in Rate, Dist, Vol Flow, and Cardiac Output in four categories of patients with cardiac dysfunction, hypertension, coronary heart disease (CHD), and hypertension & CHD at the same time.
4. Statistical methods are as follows: firstly, the independent sample *T*-test was used to compare the mean values of rate, Dist, Vol Flow, and cardiac output at different group levels. Secondly, the Mann–Whitney test was in use.

The outline of this paper is given below.

In Section 2, we described the study's design and populations. The medical record data of the patients are collected for study. Also, different methods are used to evaluate the systolic function of the left ventricle of the patient. The independent sample *T*-test and Mann–Whitney test were used to analyze the data.

In Section 3, the difference analysis of the parameters in Dist, Vol flow, and cardiac output was analyzed. Then, the descriptive statistics and difference analysis of the Rate indicators were analyzed.

In Section 4 , the significance and clinical value of the Rate will be discussed. The reasons for different outcomes of the parameters obtained by ultrasound in different cardiovascular diseases will be analyzed. And the theoretical basis for how to take advantage of artificial intelligence (AI) using Korotkoff sound will be elaborated.

In Section 5, the result section, it has been discussed that the result can provide a theoretical basis for the subsequent artificial intelligence (AI) method to predict the heart function using the Korotkoff sound, reduce the computational amount, and improve the computational speed.

## 2. Methods and Materials

In this section, methods for obtaining brachial artery vascular parameters and cardiac function indicators by using the ultrasound machine are introduced. Variables, outcome, measures, information source, bias, and statistical analysis are discussed.

### 2.1. Study Design and Patients

The Ethics Committee of the Fourth Affiliated Hospital of Zhejiang University School of Medicine review board approved this observational study, which was conducted following the principles of the Helsinki Declaration. All medical record data were collected at our medical centers.

This is an exploratory and observational study. The in-patients in the Department of Cardiovascular Medicine of the Fourth Hospital of Zhejiang University were selected from 2021.3–2021.7 without relevant intervention. Since the hospitalized patients in our center need to routinely complete the cardiac color ultrasound examination, we have no special restriction on the examination time of the patients, completely following the arrangement of HIS hospitalization system. The ultrasound examination of the brachial artery-related vascular characteristics is free and voluntary, and some precautions are informed before the test to avoid medical disputes.

The exclusion criteria for the study are as follows:

1. Rapid changes in heart rate or cardiac output are affected by tension, fatigue, excitement, full meal, fever, infection, and other inducements before the test.
2. Severe chest pain and suspected acute attack of myocardial infarction.
3. An acute hypertensive episode or hypertensive crisis with systolic pressure over 180 mmHg or diastolic pressure greater than 120 mmHg [7].
4. Coarctation of the aorta, vasculitis, pheochromocytoma, etc., whose influence on the bilateral upper limb blood pressure fluctuates greatly [8‐10].
5. Frequent arrhythmias (such as frequent atrial premature beats, atrial fibrillation, paroxysmal supraventricular tachycardia, ventricular tachycardia, etc. [11].
6. Extremely poor cardiac function, intolerance to mild activity, or severe visible pitting edema.
7. Mental patients with anxiety and panic disorder.
8. Poor compliance, i.e., those with difficulty in cooperating with the study.

### 2.2. Description of the Measurement Method

When the participants arrived at the echo lab, they needed to rest in bed in a supine position for at least 10 minutes before taking measurements. After this break, we took the measurements in a room at constant temperature (23°C–25°C) [12], which are as follows.

The overall systolic function of the left ventricle of the patient was evaluated by two professional cardiac ultrasound technicians in our hospital using the PHILIPS ultrasound instrument according to the clinical states of the patient at that time by following the established clinical guidelines [13].

Generally, the biplane method (modified Simpson) is used to measure the left ventricular volume [14]. If the image quality is good, the three-dimensional ultrasound will be applied to measure the left ventricular volume. If there is no obvious heart disease, the M-type ultrasound can be used to do [15]. From the above operation, we can obtain the left ventricular end-diastolic volume (EDV) and end-systolic volume (ESV). The PHILIPS ultrasound machine will automatically generate the LVEF and cardiac output accordingly.

After completing the above procedure, we would notice that the patient lies in a supine position with the upper limb fully exposed. Ensure that the patient is lying flat and the muscles and joints are relaxed. For the convenience of clinical measurement, all patients were measured uniformly on the right upper limb (except for patients with inconveniences in the right upper limb). Starting with the auxiliary artery, the brachial artery blood flow spectrum (Vol flow) above the bifurcated level was obtained [5]. Blood flow was calculated automatically according to the PHILIPS system's built-in algorithm, which can be summarized as Blood flow (Flow, ML·min^−1^) = Time mean flow rate (Vmean, cm·s^−1^) × Lumen cross-sectional area (S, cm^2^) [16]. To minimize the measurement errors caused by human factors, during the inspection, the probe should be perpendicular to the limb surface, and the force should be moderate to avoid pressure deflating the blood vessels and increasing the measurement error. The Doppler spectrum was obtained by slitting at the same position, and the incidence angle of ultrasound was controlled to be less than or equal to 60°. The sampling volume occupied the entire vascular lumen. The brachial artery blood flow spectrum was measured to obtain Vmean. The brachial artery short axis was explored, and the cross-sectional area was measured along the medial edge of the brachial artery lumen. All blood flow characteristics of the brachial artery were documented by a pulsed Doppler measurement.

### 2.3. Variables, Outcome Measures, Information Source, and Bias

Our primary outcome was to explore whether there would be a quantitative relationship between the brachial arterial blood flow and cardiac volume in patients (Rate = Brachial arterial blood flow/Cardiac output) and whether these two related variables would be more outstanding in patients with cardiac dysfunction.

Our secondary outcome was to know whether brachial artery diameter (Dist), blood flow (Vol Flow), and cardiac output in patients with different cardiovascular diseases have otherness.

We obtained clinical characteristics (including age, sex, height, weight, and disease) from the patient's electronic medical record system and excerpted brachial artery diameter (Dist), AREA, blood velocity (TAMV), blood flow (Vol Flow), cardiac output, and left ventricular ejection fraction (LVEF) on the ultrasound machine in the meantime [17, 18]. It is conducive to a better overall analysis.

As no reports about this hot topic exist, the results of this study cannot be tested using external databases. All the data in this paper are from the real clinical world, and no special processing is done on the data.

### 2.4. Statistical Analysis

We conducted a descriptive statistical analysis of the selected patients (*n* = 586). All measurements of the parametric type were expressed as mean ± standard deviation (*x* ± *s*). The types of nonparameter were shown as median (upper and lower quartile). The independent sample *T*-test and Mann–Whitney test were used to analyze the data [19].

In the statistical analysis of differences, the differences in rate, Dist, Vol Flow, and cardiac output in four categories of patients with cardiac dysfunction, hypertension, coronary heart disease (CHD), and hypertension & CHD were studied at the same time. LVEF, hypertension, CHD, and hypertension & CHD were considered binary nominal variables. Rate, Dist, Vol Flow, and cardiac output were continuous variables. Firstly, the independent sample *T*-test was used to compare the mean values of rate, Dist, Vol Flow, and cardiac output at different group levels. Secondly, the Mann–Whitney test was in use. The rank of the Rate, Dist, Vol Flow, and cardiac output was compared at different grouping levels. *P* < 0.05 showed that the above four indicators were statistically different, which are otherwise not.

As all the data originated from the clinical real world, we did not do any extreme processing. Data analysis was performed with the IBM SPSS Statistics 22 (La Jolla, CA, USA).

## 3. Result

In this section, 586 enrolled patients were analyzed. There were 327 patients with hypertension, 284 patients with coronary heart disease (not including patients with coronary artery sclerosis), and 172 patients with hypertension and CHD. The difference analysis of parameters in Dist, Vol Flow, and cardiac output was analyzed. Then, the descriptive statistics and difference analysis of rate indicators were analyzed.

### 3.1. Demographics, Description of the Study Population

We analyzed 586 enrolled patients. The mean age of the enrolled patients was 62.81 ± 12.48 years, of which 353 were male, accounting for 60.2%. BMI remained at 24.75 ± 3.35 on average. Forty patients in the sample had cardiac dysfunction. There were 327 patients with hypertension, 284 patients with coronary heart disease (not including patients with coronary artery sclerosis), and 172 patients with hypertension and CHD, as given in Table 1.

### 3.2. Difference Analysis of Parameters in Dist, Vol Flow, and Cardiac Output

In the patients with hypertension, coronary heart disease, or both diseases, the Dist between the different groups, regardless of the parameter (*t* = 2.352, *P* = 0.019 < 0.05) or nonparameter test (*z* = −2.496, *P* = 0.013 < 0.05), was statistically different at the level of 0.05, as shown in Table. 2.

No statistically significant difference (*P* > 0.05) was found in Vol Flow regardless of the disease population as shown in Table 3.

In patients with hypertension (*t* = 4.196, *P* < 0.05; *z* = −4.086, *P* < 0.05) or hypertension combined with CHD (*t* = 2.459, *P* = 0.014 < 0.05; *z* = −2.294, *P* = 0.022 < 0.05), there was a significant statistical difference at the level of 0.05 in cardiac output by either parametric test or nonparametric test. No statistical difference was found in patients with only CHD or cardiac dysfunction as shown in Table 4.

### 3.3. Descriptive Statistics and Difference Analysis of Rate Indicators

As observed from the table, the mean Rate is 1.23%, and the 95% confidence interval of the mean was (1.18%, 1.29%), indicating that the rate was mainly concentrated in the current numerical interval as shown in Table 5.

No significant statistical difference (*P* = 0.488) was found in the rate value regardless of the state of cardiovascular disease as shown in Table 6.

## 4. Discussion

Generally, by the observational study in the real world, our research group found that although there was no significant statistical difference (*P* = 0.488) in the rate of patients with cardiac dysfunction (Rate% = 1.16 ± 0.69), it showed a slightly decreasing trend compared with the normal group (Rate% = 1.23 ± 0.68).

From the above results of this study, we could fully analyze the value and significance of the Rate and draw the following conclusions:

(1) Patients with hypertension or coronary heart disease: the brachial artery wall diameter was significantly thicker in the hypertensive patients [Dist (cm) = 0.42 ± 0.07] whose cardiac output [CO (L/min) = 5.00 ± 1.19] was significantly higher than that in the nonhypertensive patients [CO (L/min) = 4.58 ± 1.20]. Only the wall of the brachial artery was thickened, which was demonstrated in patients with coronary heart disease [Dist (cm) = 0.41 ± 0.06].
(2) Identifying the specific signals of heart failure: why are we so interested in the Rate? The terminal stage of all cardiovascular diseases is heart failure. The AHA predicted in 2017 that by 2030, the incidence of heart failure is projected to rise by 46%, affecting more than 8 million individuals [20]. Our research group has been interested in the use of nondestructive equipment to identify the early and rapid progression of heart failure-specific signals. Heart sound equipment for recognizing heart failure patients has been put into clinical use with high specificity and sensitivity at present but is not good for popularity [21, 22].
(3) Ameliorating blood pressure measurement: with the prevalence of the blood pressure measurement, the Korotkoff sound method is coming into our sight. The Korotkoff sound is caused by the blood turbulence triggering the brachial artery wall vibration [6]. The brachial artery is a branch of systemic vessels, whose blood flow is inevitably related to cardiac output, however, whether there is a quantitative relationship between them has not been reported. If we can measure blood pressure while identifying the progression signals of heart failure, it would be a very significant achievement.
(4) Statistical analysis: regrettably, we can see that there is no significant statistical difference in rate among different cardiovascular diseases in this study. Statistically, the Rate can be regarded as a constant (Rate = 1.23%). Although we found that the mean rate of the cardiac dysfunction group (Rate = 1.16%) was slightly lower than that of the patients not moving to the cardiovascular terminal stage, no statistical significance was found. It may be because of the small sample size (*n* = 40).
(5) Factors causing no sharp changes in the cardiac output and brachial arterial blood flow as follows:
  - Similarly, the brain, as an important organ for the human body, disproportionately receives approximately 12% of the cardiac output even though it accounts for only 2% of the body's weight. Meng, L. et al. found that increasing the cardiac output will improve the cerebral blood flow in chronic heart failure patients [23].
  - The kidney blood flow is enormous, accounting for 25% of the cardiac output at rest [24]. Within a certain range of arterial blood pressure (80–160 mmHg), the renal blood flow can be kept constant via an autoregulation mechanism [25]. The disproportionate reduction in renal perfusion only occurs when the cardiac output is sharply reduced, which consequently leads to a diminished glomerular filtration rate (GFR) [26].
  - Reviewing our experimental study, after excluding the factors that cause the sharp changes in cardiac output and heart rate, we ensure that each patient completes the trial in a quiet state. Although they suffer from cardiovascular disease and possess irreversible damage, we can believe that the rate will not vary greatly with the body's compensatory regulation. As a branch of the cardiovascular system, the brachial artery is not as important as organs, such as the brain or the kidney, but it plays its role. Thus, the indicator rate has been provided with theoretical significance to some extent.
(6) Patients with hypertension and coronary heart disease reflecting the reliability of the rate: these two diseases are widely recognized as the leading causes of death in cardiovascular patients [20]. Our research team analyzed the data from the lateral perspective of the patients with hypertension, coronary heart disease, or both.

### 4.1. Patients with Hypertension

Let's retrospect the patients with hypertension (*n* = 327). Firstly, the variable Dist [Dist (cm) = 0.42 ± 0.07] between the different groups, regardless of the parameter or nonparameter test, was statistically different at the level of 0.05 (*P* < 0.05), so is the cardiac output [CO (L/min) = 5.00 ± 1.19]. However, there was no statistical difference in Vol Flow. Current research on hypertension has focused on two aspects: vascular resistance and arteriole [27]. For all we know, under the impact of a prolonged state of high blood flow, the musculature of the blood vessel wall will degenerate, eventually losing its toughness and being replaced with stiffer fibrous connective tissue. If no drug intervention or left untreated, the body's activated RAS axis will allow the body to adapt to the state of decompensation of high pressure, forming positive feedback, and it eventually deteriorates the cardiac function, moving to the final stage of cardiovascular heart failure [28–31].

As to why there was no statistical difference in Vol Flow, some differences in the plane may be obtained by different ultrasonic sections, and unlike the wall diameter, the flow velocity is not objective and authentic, and it will be interfered with by numerous factors [13]. The specific mechanism remains to be explored. To sum up, the vascular resistance remodeling of arterioles is a marker of the pathophysiology of hypertension, and the clinical data we acquired are reliable and credible [32].

### 4.2. Patients with Cardiovascular Disease

The statistically significant factors for coronary heart disease are given as follows:

- To examine the outcomes for patients suffering from coronary heart disease (*n* = 302). In both parametric test and nonparametric test, the Dist [Dist (cm) = 0.41 ± 0.06] of patients with coronary heart disease was statistically significant (*P* < 0.05), while Vol Flow and Cardiac Output were not.
- To make the data more salient, we did not include patients with coronary atherosclerosis as coronary artery disease is diagnosed only when the degree of coronary artery obstruction is greater than 50% [33]. The process of atherosclerosis begins as early as childhood [34], and coronary heart disease is a more serious state of coronary atherosclerosis. It is not difficult to deduce that our data set is reliant and reliable.
- As to why there was no significant statistical difference between the other two indicators, we speculated that the long-term self-regulation of patients suffering from coronary heart disease would increase the collateral circulation of the heart, thus allowing the body to adapt to the pathological state so that there is no significant difference compared with the nondiseased population.

Combined with the above analysis, the statistical results of hypertension and CHD at the same time showed significant statistical differences in Dist and cardiac output, however, there were no statistical differences in Vol Flow. From this, we can boldly speculate that hypertension may be the leading factor causing the increased cardiac output [32].

BMI was in the different analyses: concretely, we were unable to define a meaningful critical interval for BMI. A decline in BMI was independently correlated to death in patients with myocardial infarction, left ventricular systolic insufficiency, and heart failure according to the existing clinical studies [35]. Although these associations may reflect some patient conditions, causality cannot be inferred.

The theoretical basis for taking advantage of artificial intelligence (AI) using Korotkoff sound: what can we do with the Rate value? Our research group has been working on the nondestructive monitoring of diseases. Today, with the prevalence of artificial intelligence technology (AI) and the widespread popularity of sphygmomanometer measurement, we can make an intelligent sphygmomanometer based on the Korotkoff sound, which provides us with the possibility of early identification of progressive signals of heart failure [36]. Although there was no significant statistical difference in rate in the population of cardiac dysfunction (probably due to the limitation of sample size), there was still a downward trend in rate compared with patients with normal cardiac function. To a large extent, it can reduce the amount of computation for our machines. In addition, the Dist of patients with hypertension and coronary heart disease showed significant differences, which is bound to produce qualitative alternatives in the acoustic characteristics of blood flow impacting the tube wall. To a certain extent, the above principles can be the believed biological traits.

This study had some unavoidable limitations. Considering the economic benefits of the hospital and the pressure on the staff, we only conducted free brachial blood flow measurements for 4 months. It was done in patients who developed the related cardiovascular disease but not in a completely normal healthy population or in patients who did not develop cardiovascular disease. As no one has explored this hot topic at present, the external database cannot be used to verify the experimental research results. Because of technical and conditional limitations, it is impossible to measure cardiac output and blood flow of the brachial artery at the same time. The current season is not the peak morbidity for heart failure patients, and hence, the sample size of patients with cardiac dysfunction is very limited. Based on the above characteristics, it is not possible to follow-up with the above patients actively in a short time to observe the difference of each indicator.

## 5. Conclusions

In conclusion, we have sufficient reasons to believe that the Rate is a constant of 1.23% approximately, and the mean 95% CI was (1.18%, 1.29%) before the cardiovascular disease reached the terminal stage. Though the rate in the population of cardiac dysfunction (1.16% ± 0.69) is not significantly different, this value tends to decrease relative to the normal population. The result can provide a theoretical basis for the subsequent artificial intelligence (AI) method to predict heart function by the Korotkoff sound, reduce the computational amount, and improve the computational speed.

Also, the results of this observational study indirectly prove that the pathological thickening of the peripheral vascular arterioles occurs in hypertension [Dist (cm) = 0.42 ± 0.07] and coronary heart disease [Dist (cm) = 0.41 ± 0.06]. The patients suffering from hypertension often show higher cardiac output [CO (L/min) = 5.00 ± 1.19].

## Figures and Tables

**Table 1:** Characteristics of participants.

Categorical variables			Count/mean	*N*%/std.
Age			62.79	12.48
Gender	Male		353	60.24%
	Female		233	39.76%
	Total		586	100.00%
BMI			24.75	3.35
Dist (cm)			0.40	0.07
Area (cm^2^)			0.1400	0.1489
TAMV (cm/s)			7.73	4.55
Vol Flow (cc/min)			58.66	35.83
Cardiac output (L/min)			4.81	1.21
Cardiac disfunction		Normal (LVEF ≥ 50%) [15, 16]	546	93.17%
		Abnormal (LVEF < 50%)	40	6.83%
		Total	586	100.00%
Hypertension		No	259	44.20%
		Yes	327	55.80%
		Total	586	100.00%
Coronary heart disease (CHD)		No	302	51.54%
		Yes	284	48.46%
		Total	586	100.00%
Hypertension & CHD		No	414	70.65%
		Yes	172	29.35%
		Total	586	100.00%

**Table 2:** Difference analysis on Dist.

Dist (cm)		*N*	*T*-test						NPar tests		
			Mean ± SD	Levene's test		*t*-test			Median (Q1, Q3)	Z	*P*
Item	Level			*F*	*P*	T	df	*P*			
Cardiac disfunction	Abnormal	40	0.416 ± 0.0837	1.376	0.241	1.154	584.000	0.249	0.406 (0.3569, 0.464)	−0.858	0.391
	Normal	546	0.4028 ± 0.0692						0.401 (0.3549, 0.453)		

Hypertension	Yes	327	0.4167 ± 0.0718	1.842	0.175	5.134	584.000	<0.001	0.4109 (0.3679, 0.464)	−4.701	<0.001
	No	259	0.3873 ± 0.0649						0.389 (0.3469, 0.432)		

Coronary heart disease (CHD)	Yes	284	0.4106 ± 0.0638	8.348	0.004	2.352	577.672	0.019	0.4055 (0.3679, 0.455)	−2.496	0.013
	No	302	0.3971 ± 0.0754						0.389 (0.3449, 0.447)		

Hypertension & CHD	Yes	172	0.4207 ± 0.0648	2.275	0.132	3.815	584.000	<0.001	0.4219 (0.373, 0.464)	−3.804	<0.001
	No	414	0.3966 ± 0.0714						0.39 (0.3469, 0.445)		

**Table 3:** Difference analysis on Vol Flow.

Vol Flow (cc/min)		*N*	*T*-test						NPar tests		
			Mean ± SD	Levene's test		*t*-test			Median (Q1, Q3)	Z	*P*
Item	Level			*F*	*P*	t	df	*P*			
Cardiac disfunction	Abnormal	40	51.3098 ± 35.0009	<0.001	0.994	−1.346	584.000	0.179	38.8 (28.2, 68.75)	−1.725	0.085
	Normal	546	59.2037 ± 35.8642						50.4 (33.5, 76.2)		

Hypertension	Yes	327	60.5759 ± 35.5742	0.060	0.807	1.452	584.000	0.147	51.2 (36.1, 77.1)	−1.929	0.054
	No	259	56.2522 ± 36.0791						48.4 (30.2, 73.9)		

Coronary heart disease (CHD)	Yes	284	59.83 ± 36.2618	0.086	0.770	0.763	584.000	0.446	50.85 (35.15, 75.05)	−1.131	0.258
	No	302	57.5693 ± 35.4484						49.35 (30.8, 76.1)		

Hypertension & CHD	Yes	172	60.749 ± 34.6142	0.536	0.464	0.907	584.000	0.365	52.1 (36.55, 76.75)	−1.566	0.117
	No	414	57.7991 ± 36.3319						49.1 (30.9, 75.3)		

**Table 4:** Difference analysis on cardiac output.

Cardiac Output (L/min)		*N*	*T*-test						NPar tests		
			Mean ± SD	Levene's test		*t*-test			Median (Q1, Q3)	*Z*	*P*
Item	Level			*F*	*P*	*T*	df	*P*			
Cardiac disfunction	Abnormal	40	4.5477 ± 1.5555	8.490	0.004	−1.138	42.359	0.261	4.63 (3.345, 5.655)	−1.112	0.266
	Normal	546	4.8335 ± 1.1812						4.775 (4.01, 5.56)		

Hypertension	Yes	327	4.9982 ± 1.192	0.049	0.825	4.196	584.000	<0.001	4.89 (4.15, 5.72)	−4.086	<0.001
	No	259	4.5814 ± 1.1966						4.56 (3.81, 5.22)		

Coronary heart disease (CHD)	Yes	284	4.8074 ± 1.1893	0.847	0.358	−0.127	584.000	0.899	4.695 (3.985, 5.495)	−0.605	0.545
	No	302	4.8201 ± 1.2328						4.805 (3.94, 5.66)		

Hypertension & CHD	Yes	172	5.004 ± 1.1378	1.356	0.245	2.459	584.000	0.014	4.86 (4.155, 5.625)	−2.294	0.022
	No	414	4.735 ± 1.2327						4.7 (3.85, 5.53)		

**Table 5:** Descriptive statistics about Rate.

			Statistic	Std. error
Rate	Mean		1.2310	0.02826
	95% confidence interval for mean	Lower bound	1.1755	
		Upper bound	1.2865	
	5% trimmed mean		1.1849	
	Median		1.1074	
	Variance		0.4650	
	Std. deviation		0.6818	
	Minimum		0.0048	
	Maximum		5.3608	
	Range		5.3560	
	Interquartile range		0.8650	
	Skewness		1.219	0.101
	Kurtosis		2.788	0.202

**Table 6:** Descriptive statistics about Rate.

Rate		*N*	*T*-test						NPar tests		
			Mean ± SD	Levene's test		*t*-test			Median (Q1, Q3)	*Z*	*P*
Item	Level			*F*	*P*	*t*	df	*P*			
Cardiac disfunction	Abnormal	40	1.1606 ± 0.6917	0.277	0.599	−0.695	584	0.488	1.0454 (0.6447, 1.704)	−0.843	0.399
	Normal	546	1.2384 ± 0.6824						1.1221 (0.7377, 1.5965)		

Hypertension	Yes	327	1.2323 ± 0.6668	1.254	0.263	−0.028	584	0.977	1.1471 (0.736, 1.5989)	−0.426	0.670
	No	259	1.234 ± 0.7037						1.0762 (0.7292, 1.6346)		

Coronary heart disease (CHD)	Yes	284	1.2593 ± 0.6956	0.045	0.831	0.903	584	0.367	1.1371 (0.7676, 1.641)	−1.049	0.294
	No	302	1.2084 ± 0.6706						1.0581 (0.7038, 1.5938)		

Hypertension & CHD	Yes	172	1.2362 ± 0.6744	1.122	0.290	0.072	584	0.942	1.1404 (0.7676, 1.5961)	−0.426	0.670
	No	414	1.2317 ± 0.687						1.0968 (0.7235, 1.6027)		

## Data Availability

The datasets used and analyzed during the current study are available from the corresponding author upon reasonable request.
